The article "Outcomes and Disease Spectrum of LBW Neonates in a Secondary Health Facility" was published in 2022. Journal: J Healthc Eng.

# Outcomes and Disease Spectrum of LBW Neonates in a Secondary Health Facility

**DOI:** 10.1155/2022/9974636

**Published:** 2022-01-27

**Authors:** Rosena Olubanke Oluwafemi, Femi Peter Adesina, Adebola Olutoyin Hassan

**Affiliations:** ^1^Paediatrics Department, Mother and Child Hospital, Akure, Nigeria; ^2^Department of Biology, Federal University of Technology Akure, Akure, Nigeria; ^3^Family Health Department, UNICEF, Abuja, Nigeria

## Abstract

Globally, 30 million low birth weight (LBW) babies are born every year and 95% of them are from developing countries. LBW neonates are at a high risk of mortality, morbidity, and long-term disability. The objective of this study is to investigate outcomes and disease spectrum among low birth weight neonates. This is a prospective, observational study conducted on 540 neonates admitted in the Mother and Child Hospital, Akure, Ondo State, Nigeria, from 2017 to 2018. Questionnaire, interview, clinical, and diagnostic procedures were used as research tools. There were 137 low birth weight (LBW) neonates, with the mean mothers' age of 31.92 ± 6.60. Of the 540 neonates, 69 (50.4%) and 68 (49.6%) were term and preterm, respectively. There were 64 female neonates (46.7%) and 73 male neonates (53.3%). The mean weight of the neonates was 1.82 ± 0.44 kg, and mean number of days on admission was 6.42 ± 6.75 days. Neonatal sepsis (NNS) was the highest morbidity 51 (37.2%) among the LBW neonates, followed by prematurity 47 (34.4%) and neonatal jaundice (NNJ) 18 (13.1%). Sex (***χ***^**2**^ = 3.584, *p*=0.310), mode of delivery (***χ***^**2**^ = 4.669, *p*=0.198), and gestational age (***χ***^**2**^ = 3.904, *p*=0.272) were not a significant determinant of outcome among LBW neonates. Men were 2.36 times more likely to be preterm (OR = 2.36, 95% CL = 1.01–5.54, *p*=0.048) among LBW neonates. Outcomes of LBW neonates who were delivered by SVD were not significant compared to preterm delivered by CS (OR = 0.46, 95% CL = 0.13–1.65, *p*=0.096). Sixty percent (60%) of the mothers had Prolonged Rupture of Membranes (PROM). Morbidities such as hypothermia (72.2%), apnoea (63.6%), haemorrhagic disease of the newborn (HDN) (66.7%), and respiratory distress syndrome (RDS) (66.7%) were more observed with preterm LBW neonates. Importance of qualitative antenatal care (ANC) should be emphasized; anticipation and prevention of LBW births can help mitigate some of the problems they are prone to.

## 1. Introduction

Neonate's birth weight can be categorized to be low birth weight (<2,500 g), normal birth weight (2,500 to 4,000 g), and high birth weight (>4,000 g) [1]. Low birth and high birth weight are called abnormal birth weights (ABW) [2, 3]. Two major determinants of birth weight include the gestational age and intrauterine growth rate [4] and this means low birth weight is either as a result of prematurity (<37 completed weeks), intrauterine growth restriction, or both [5], the latter being primarily as a result of intrauterine malnutrition from altered placental circulation.

Globally, 30 million of low birth weight (LBW) occurs every year and 95% of them are from developing countries [6, 7]. Low birth weight is a major contributory factor to neonatal ill health and by extension child morbidity, mortality, and disability [8–10]. A cohort study on cognitive abilities, educational progress, and behavioral problems in very low birth infants followed up for 8 years showed they all lagged behind the controls (birth weight >2499 g) [11]. By WHO definition, low birth weight is a birth weight of <2,500 g [12]. Low birth is further classified into extremely low birth weight (≤1,000 g) and very low birth weight (<1,500 g) [13].

Several factors have been associated with low birth weight though not necessarily in isolation. Maternal factors could be responsible for this, such as congenital malformations of the uterus, prenatal malnutrition and lifestyle, maternal illnesses such as hypertension or diabetes in pregnancy, infection with bacterial vaginosis, malaria, and flu. Race, maternal age, socioeconomic factors, and parity are also contributory factors [14–16]. Incidence of low birth weight seems to be higher in teenage mothers, Blacks, and Asians.

Obstetric factors such as previous stillbirth, short birth interval, inadequate prenatal care, placenta previa, and abruption [17] could also be responsible. A clinical trial showed a 15% reduction in incidence of LBW when mothers were immunized with influenza vaccines [18]. Socioeconomic factors also play a critical role in low birth weight [19] as evidenced by a study in Iceland, which showed a significant rise in the incidence of preterm delivery after the severe economic decline affected young women who had no jobs especially in their 3^rd^ trimesters [20].

The outcomes of low birth weight are also dependent on other factors such as an enabling environment with adequate and effective perinatal and neonatal care, skilled birth attendants, and appropriate equipment and technological advancement in the care of such special cohort of newborns. In developed countries, survival rates of LBWs have improved due to the requisite skills and availability of appropriate equipment to support the low birth baby. Though the requisite skills and equipment might be lacking in the developing countries, the introduction of Kangaroo Mother Care has improved the survival rates in LBWs with comparable significantly better rates with the conventional methods [21].

In Africa, 5.7 million of LBW neonates are recorded every year [22]. In 2018, Nigeria recorded a prevalence of 7% LBW, with 7.5% of it in the urban and 6.9% of it in the rural [23]. The study on outcome of LBW is very important to ascertain improvement in maternal and neonatal health care services. Therefore, the objective of this study is to determine the outcome of LBW infants either born or referred to the Mother and Child Hospital, Akure, Ondo State.

## 2. Material and Methods

### 2.1. Study Area

The study was carried out at the Mother and Child Hospital, Akure (MCHA), a modern secondary public health facility providing specialized free health services to the state capital and surrounding communities. It also serves as a referral care center for other government, private, and missionary hospitals. The Mother and Child Hospital Akure is located in the city of Akure, the capital city of Ondo State. Ondo State lies between latitudes 5°45' and 7°52'N and longitudes 4°20' and 6°5'E. Its land area is about 15,500 square kilometers. Ondo State has an estimated population of 5,372,477, with over 1,715,820 female inhabitants base on projection from the 2006 Nigeria national population.

### 2.2. Study Design and Population

This is an observational prospective study conducted on 540 neonatal admission for one year (May 2017 to April 2018). All the births were studied till either discharged from the hospital or inadvertent death.

### 2.3. Data Collection

A well-structured questionnaire was used for the collection of the socio-demography data of the baby's father and mother. Before applying the questionnaire to the target population, pretesting was carried out with twenty (20) women who are not part of the study group; this was to ascertain simplicity and the objective accuracy. A well-trained nurse and medical assistants were recruited to assist in administering the questionnaires and to conduct interviews for the parents and also in taking clinical and diagnostic data. Information collected included mother and father's age, educational level, occupation, marital status, antenatal visit, gestational age, neonate's birth weight, place of delivery, and days on admission was also monitored.

Each baby was weighed using the *RGZ-20* weighing scale. The scale records weights in grams to the nearest 25 g. It was adjusted for zero error before each reading. Other measures taken to ensure reliability of results included weekly standardization of the weighing scale, using known weights.

Physical examination and laboratory findings as well as clinical history were done to ascertain complications and it was carried out by the attending neonatologist. Some of the conditions were defined as follows:

- Apnoea defined as cessation of breathing lasting for 20 seconds or more, associated with bradycardia or cyanosis and needing resuscitation
- Neonatal sepsis defined as clinical signs and symptoms suggestive of neonatal infections positive laboratory indices and multiple organ involvement
- Neonatal jaundice is a yellowish discoloration of the sclera and skin and serum bilirubin up to 5 mg/dl
- Severe birth asphyxia defined as an APGAR score of 5 or less at 5 minutes and with neurological manifestations or babies with multiple organ involvement
- Hypoglycemia defined as random blood glucose of <50 mg/dl
- Anemia defined as hemoglobin level <10 g/dl
- Hypothermia defined as a rectal temperature of <35°C
- Failure-to-thrive (FTT) was used to describe inadequate growth, failure to gain weight or height, and the inability of the baby to maintain growth according to the standard growth chart; it is a sign of multiple problems as well as undernutrition

### 2.4. Inclusion Criteria

The enrollment was based on any live birth <2,500 g in MCHA and neonates transferred in.

### 2.5. Exclusion Criteria

The excluded were children whose parents did not give their consent, babies with congenital abnormalities, and stillbirths.

### 2.6. Ethical Clearance

Ethical procedures were followed obtaining permission for the study from the Research and Ethics Committee in the MCHA. Informed consent was obtained from parents of participants.

### 2.7. Data Analysis

Statistical analysis was carried on the collected data, using SPSS (version 21.0), and graphs were generated using Microsoft Excel. The chi-squared test was done to determine if gestational age and outcome of admission depend on mother's sociodemographic variables. The logistic regression procedure was used to determine the risk factors of LBW neonates in the studied area. Level of significance for this study is put at *p* < 0.05.

## 3. Results

Table 1 shows the socio-demographic data of the neonates' parents in the MCHA. There were 137 low birth weight (LBW) neonates. More than half 87 (63.5%) of the mothers were of age 30–39 years, with the mean age of 31.92 ± 6.60. Majority of the mothers were self-employed 80 (58.4%), married 133 (97.1%), and almost half 66 (48.1%) of the mothers had tertiary education.

Table 2 shows that the mean age ± SD at presentation is 6 ± 7.7 days. Almost the same number of term 69 (50.4%) and preterm 68 (49.6%) was recorded. There were 64 female babies (46.7%) and 73 male babies (53.3%). The majority of LBW neonates were delivered by Spontaneous Vertex Delivery 116 (84.7%). Also, the mean neonate's weight was 1.82 ± 0.44 kg and mean of days on admission was 6.42 ± 6.75 days. Higher proportion of their mothers attended antenatal clinic 117 (85.4%), before delivery.

Figure 1 shows that 100 (73.0%) of the LBW neonates were discharged alive, 8 (5.8%) were discharged against medical advice (DAMA), 9 (6.6%) were referred, and 20 (14.6%) of the LBW neonates died.

The disease spectrum of LBW neonates is shown in Table 3. Neonatal sepsis (NNS) had highest occurrence 79 (57.7%) among the LBW neonates, followed by neonatal jaundice (NNJ) 48 (35.5%), prematurity 47 (34.4%), PROM 30 (21.9%), Apnoea 22 (16.1%), hypothermia 18 (13.1%), respiratory distress syndrome 15 (10.9%), hypoglycemia 10 (7.3%), and haemorrhagic disease of the new born 3 (2.2%).

Sex (***χ***^**2**^ = 3.584, *p*=0.310), method of delivery (***χ***^**2**^ = 4.669, *p*=0.198), and gestational age (***χ***^**2**^ = 3.904, *p*=0.272) are not a significant determinant of outcome among LBW neonates, except neonate's weight (***χ***^**2**^ = 21.216, *p*=0.002) (Table 4). In Table 5, the mother's age 30–39 years and 40–49 years were 1.82 and 2.39 times likely to deliver preterm babies, respectively, than 20–29 years of age. Neonates' sex was significantly associated with gestational age (OR = 2.36, 95% CL = 1.01–5.54, *p*=0.048) among LBW neonates. Also, the neonates' gestational age (*χ*^2^ = 32.428, *p*=0.001) significantly determined their weight.

PROM (60%), hypothermia (72.2%), apnoea (63.6%), haemorrhagic disease-HDN (66.7%), and respiratory distress syndrome-RDS (66.7%) were more observed with preterm LBW neonates (Figure 2). In Figure 3, diseases that are more recorded with male LBW neonates were PROM (56.7%), hypothermia (66.7%), NNS (51.9%), and RDS (60.0%). Hypoglycemia (60.0%), apnoea (54.5%), HDN (66.7%), RVS (66.7%), and rhesus isoimmunization (100%) were common with female LBW neonates.

## 4. Discussion

Within the period of study, 540 neonates were admitted and majority of the neonates (75.9%) were referred from other government hospitals to MCHA. The incidence of low birth weight (LBW) among the neonates in the current study was 25.37%. This figure is higher than the reports of 2.6% in the 45 months of study from Enugu, southeast, and Nigeria [10], 6.3% from Nsukka and Calabar [16], 8.3% from Port-Harcourt [24], and 15.7% from Maiduguri [25]. Likewise, it is higher than report of 12.3% from Kenya in a cross-sectional analytical study conducted by Muchemi et al. [13] in Olkalou District Hospital and 14.6% prevalence from a hospital-based observational study in Ethiopia by Melkamu et al. [17]. Higher incidence recorded in this study may be due to the fact that majority of the babies were referred in, MCHA being a major referral center and highly specialized for maternal and under-5 care for other hospitals around the region. Again, the disparity in LBW prevalence across countries may be due to economic and environmental factors. According to Lee et al. [26], 14% of neonates in low-income countries were stated to have low birth weight (<2,500 g), with many of them born preterm. From the datasets of birth record collected by Fayehun and Asa [1] and from Nigeria Demographic and Health Survey (NDHS), the prevalence of LBW in urban areas was 18.3% between 2013 and 2018. Furthermore, the incidence of preterm in the current study was 49.6%, which is comparatively higher than the previous report of 15.4% reported from the same center (MCHA), in 2016 [27] and of 18.5% from Lagos [4] among babies delivered. The incidence of preterm was however lower than report of 90% from Enugu [10] and 68% from Port-Harcourt [24].

In 2019, Melkamu et al. [17] reported factors that influenced LBW delivery to be mother's socio-demography status such as low maternal age, low level of education, and occupation (stressful job). Other factors identified by other researchers include maternal weight less than 50 kg, gestational age of baby (<37 weeks), maternal anemia (hemoglobin less than 10 gm/dl), maternal illness, multiple pregnancy, physical violence, exposure to environmental pollutants (pesticides), poor support from the husband or family, poverty, and nutrition (undernutrition, smoking of tobacco, alcohol ingestion, or iron deficiency) [4, 13, 17, 28–30]. Meanwhile, in the current study, it was not significantly evident that mothers' age contributed to LBW neonates, but it was observed that most of LBW neonates' mothers were between 30 and 39 years old, with a mean age of 31.92 ± 6.60. Goisis et al. [15] reported that there was no association between advanced maternal age and low birth weight or preterm among Finnish mothers and in contrast, Alehegn et al. [31] noted that age 40 and above were more prone to have LBW newborns compared to a maternal age of 30–34 years. On the other hand, the mother's age less than 19 years old was revealed to be more of risk of delivering LBW babies because their reproductive system might not have fully developed and also likely due to economic deficiency and self-neglect [29, 32] in terms of health care. The difference on this view of maternal age and LBW may be due to other factors that may influence LBW but not observed in each study.

Mothers with secondary and tertiary education were 0.88 and 0.66 time, respectively, less likely to experience low birth weight delivery than mothers with lower educational levels. In accordance with this study, reports by Maznah et al. [33] on 2013 Nigeria Demographic and Health Survey show that maternal education has a significant association with birth weight of their infants. Silvestrin et al. [34] also opined that having a higher education serves as protection against LBW delivery than having a lower education. Higher education increases the mothers' level of awareness and understanding, thereby helps in safeguarding mothers from careless attitude about their health. In contrary, some other researchers revealed from their study that a mother's level of education has no significant effect on birth weight [35, 36].

Also, in the current study, majority of the mothers of the low birth weight babies had ANC; this is contrary to a study by Yaya et al. [37] where participants who do not receive ANC had a higher odds of a low birth weight or preterm baby. In 2016, WHO made an adjustment on the minimum number of ANC contacts recommended for pregnant woman from 4 times to 8 times [38]. It is expected that during ANC periods, risk for delivery should be identified, prevented, and managed [39]. Analysis of community-based study in seven Western provinces of China by Ref. [40] reported that mothers who did not make up to five ANC contacts during pregnancy had a higher risk of LBW babies than mothers who had it and also added the importance of the ANC to be an ultimate contributor to avoid LBW and other complications, through early detection that leads to timely diagnoses and therapeutic intervention. The disagreement of this study to other studies concerning the ANC in relation to LBW may be due to the fact that this study did not examine the number of ANC received by neonate's mothers. On the other hands, mothers who attested to taking ANC might not have had the minimum required ANC contacts or might not have followed recommendations made during ANC session due to economic or financial constraints. Components of antenatal care (services render) differ from place to place [41]. LBW delivery is also possible because some of the mothers did not enroll in appropriate health facilities as many were captured to have delivered their babies at Church/mission (7.3%), home or traditional home (8.0%), and farm (3.6%). Likewise, Branco da Fonseca et al. [42] affirmed that not having adequate number of antenatal care visits is associated with low birth weight.

Furthermore, working mothers were 5 times more likely prone to have a low birth weight infant than the housekeeper and self-employed mothers [43, 44]. In the low-economy countries where government work is not readily available or mother's education cannot secure a good job, in order for mothers to assist their husband or meet up with standard of living, they engaged in strenuous work (even when pregnant) like standing for long hours, hawking, lifting objects, and physical hard works. These strenuous works have been associated with outcomes (preterm and LBW) and complications in the neonates [45]. Working more than 8 hours per week may lead to low birth weight [44].

Extreme low birth weight (ELBW) neonates recorded in this study were 100% preterm, while the very low birth weight (VLBW) was 95.7% preterm. This shows that the low birth weight is strongly associated with gestational age. Several other researchers have also affirmed it [4, 30, 35, 46, 47].

There was a slightly higher number (53.3%) of a male LBW neonate in this study. The binary logistic analysis further revealed that male babies were 2.36 times preterm than their female counterpart. Several researchers have corroborated this finding [48–50]. Reports by Kramer pointed out that the male genes are a significant contributing factor to being born as a low birth weight [51]. While other evidence suggested that male preterm birth is due to hormonal action, more inflammatory maker in the placental bed of the male fetus and that mothers of male fetuses showed more adverse reactions to these markers and these mothers are more prone to complications [52–54]. In contrast, female neonates were 1.62 times more likely to be born with low weights and preterm in a study conducted by Melkamu et al. [17]. However, there were a higher number of deaths (60%) recorded among female LBW neonates. RVS, rhesus isoimmunization, HDN, apnoea, and hypoglycemia were complications that were more associated to female LBW neonates in this study.

The immediate outcomes of the LBWs showed that 80.6% of babies in the range of 1500–2499 g were discharged alive from the hospital and are in keeping with the study done in National Institute of Child Health by the American Association of Pediatricians where it was proven that outcomes improved significantly with birth weights. In addition to this, Lemons et al. [21] recorded 97% discharge among 1251–1500 g and 54% among the 501–750 g. In the current study, 80.6% of the LBW were discharged alive and only 1.6% died while there was 50% survival and 50% deaths among the babies whose weight ranged between 600 and 999 g. This is an improvement in survival rate of the ELBW compared to 70.6% mortality in the previous study conducted earlier on in the same center [27].

In the current study, 6.6% of the studied LBW neonates were later referred to the surgical unit for surgical interventions. Overall, there was 14.6% mortality. Neonatal death recorded in this study is very low compared to 30% death reported by Chidiebere et al. [10] from a health facility in South East of Nigeria. Total discharged was 73.0% of LBW neonates admitted, and mean of days on admission of LBW neonates recruited was 6.42 ± 6.72. There were 2 of them that spent more than 22 days on admission. This higher number of discharge was also reported by Koc et al. [55], where 3381 (77.99%) VLBW infants were discharged out of 4335 VLBW infants admitted in neonatal intensive care units (NICUs) in Turkey, and also recorded 22% mortality during their study. Neonates and infant's death have been associated with low birth weight, and according to Elflein [56], 16.5% of all infant deaths in the United States is as a result of LBW.

Among the disease spectrum associated with LBW babies, neonatal sepsis ranked highest at 57.7% in the current study. This is not surprising; many of the babies were born in unusual places such as Church, home, and farm. Essential newborn care (drying, warming, immediate and exclusive breastfeeding, hygiene, and cord care) as well as basic care for feeding support, infection control, and breathing support which can make the difference between life and death for small babies cannot be found in these places. The current study also reported morbidities such as hypoglycemia (7.3%), hypothermia (13.1%), and apnoea (16.1%). LBW newborns are particularly susceptible to heat loss immediately after birth as a result of a high body surface area–to–body weight ratio, decreased brown fat stores, nonkeratinized skin, and decreased glycogen store [10]. All these happen as a cascade leading to hypoglycemia and apnoea coupled with immaturity of the brain and multiple ischemic brain injuries caused by recurrent hypoxic and bradycardiac spells. These have also been reported by other researchers [10, 55, 57–59]. This is unlike the study by Lemons et al. [21] where acute pulmonary disease was the highest comorbidity among the LBW babies. These differences could be due to environmental factors and a probable infection prevention and control practices.

## 5. Conclusions

The number of dead neonates in this study is still of concern, and amelioration of survival rate of low birth weight babies is important in our society. More emphasis should be placed on the importance of qualitative antenatal care (ANC) for the pregnant women. This will foster education among women for early prevention, detection, and better management and consequently better outcomes of LBW neonates.

## Figures and Tables

**Figure 1:** Outcome of LBW neonates in MCHA.

**Figure 2:** Diseases associated with gestational age.

**Figure 3:** Diseases associated with neonates' sex.

**Table 1:** Socio-demographic data of the neonates' parents.

Variable		Frequency	Percent	Mean (SD)
Mother's age	20–29 years	42	30.7	31.92 (6.60)
	30–39 years	87	63.5	
	40–49 years	8	5.8	

Mother's occupation	Self-employed	80	58.4	
	Student	8	5.8	
	Employed	35	25.5	
	Unemployed	14	10.3	

Marital status	Married	133	97.1	
	Unmarried	3	2.2	
	Separated	1	0.7	

Mother's education	Primary	12	8.8	
	Secondary	59	43.1	
	Tertiary	66	48.1	

Father's age	20–29 years	9	6.6	37.18 (5.81)
	30–39 years	74	54.0	
	40–49 years	51	37.2	
	≥50 years	3	2.2	

Father's occupation	Self-employed	68	49.6	
	Student	2	1.5	
	Employed	58	42.3	
	Unemployed	9	6.6	

Father's education	Primary	9	6.6	
	Secondary	53	38.7	
	Tertiary	75	54.7	

**SD**: standard deviation.

**Table 2:** Demographic and clinical status of LBW neonates in MCHA.

Variable		Frequency	Percentage	Mean (SD)
Age at presentation	1–7 days	101	73.7	6.11 (7.81)
	8–14 days	16	11.7	
	15–21 days	15	11.0	
	22–28 days	4	2.9	
	>28 days	1	0.7	

Gestational age	Term	69	50.4	
	Preterm	68	49.6	

Sex	Female	64	46.7	
	Male	73	53.3	

Mode of delivery	CS	21	15.3	
	SVD	116	84.7	

Neonate's weight (g)	600–<1000	6	4.4	1.82 (0.44)
	1000–1499	23	16.8	
	1500–2499	108	78.8	

Days on admission	<8 days	101	73.7	6.42 (6.75)
	8–14 days	23	16.8	
	15–21 days	11	8.0	
	>22 days	2	1.5	

Place of delivery	Government hospital	104	76.0	
	Private hospital	7	5.1	
	Home	11	8.0	
	Church/mission	10	7.3	
	Farm	5	3.6	

Antenatal care	Yes	117	85.4	
	No	20	14.6	

**Table 3:** Disease spectrum of LBW neonates in MCHA.

Problems on admission	Frequency	Percentages
Neonatal sepsis	79	57.7
Neonatal jaundice	48	35.5
Prematurity	47	34.3
Prolonged Rupture of Membranes	30	21.9
Apnoea	22	16.1
Hypothermia	18	13.1
Respiratory distress syndrome	15	10.9
Hypoglycemia	10	7.3
SBA/HIE	10	7.3
Others	6	4.4
Haemorrhagic disease of the newborn	3	2.2
Retroviral disease	3	2.2
Neonatal tetanus	2	1.5
Anorectal agenesis	1	0.7
Failure-to-Thrive	1	0.7
Rhesus isoimmunization	1	0.7
Dehydration fever	1	0.7

Others: postmaturity, aspiration pneumonitis, SBA: severe birth asphyxia, HIE: hypoxic ischemic encephalopathy LBW: low birth weight, MCHA: Mother and Child Hospital.

**Table 4:** Determinant of outcome among LBW neonates in MCHA.

Variables		Outcome				*χ* ^2^	*p* value
		Discharge	DAMA	Referred	Dead		
Sex	Female	47 (73.40%)	2 (3.10%)	3 (4.70%)	12 (18.8%)	3.584	0.310
	Male	53 (72.60%)	6 (8.20%)	6 (8.20%)	8 (11.10%)		
Gestational age	Term	55 (79.70%)	2 (2.90%)	4 (5.80%)	8 (11.60%)	3.904	0.272
	Preterm	45 (66.20%)	6 (8.80%)	5 (7.40%)	12 (17.60%)		
Mode of delivery	CS	15 (71.40%)	3 (14.30%)	0 (0.00%)	3 (14.30%)	4.669	0.198
	SVD	85 (73.30%)	5 (4.30%)	9 (7.8%)	17 (14.70%)		
Neonate's weight (g)	600–999	3 (50.00%)	0 (0.00%)	0 (0.00%)	3 (50.00%)	21.216	0.002^*∗*^
	1000–1499	10 (43.50%)	2 (8.70%)	3 (13.0%)	8 (34.80%)		
	1500–2499	87 (80.60%)	6 (5.60%)	6 (5.60%)	9 (8.30%)		

*χ* ^2^ **:** chi square, ^*∗*^: significant (*p* < 0.05).

**Table 5:** Determinant of gestational age among LBW neonates in MCHA.

Variables		Gestational age		*χ* ^2^	*p* value	OR (95% C. I. for EXP (B))
		Term	Preterm			
Mother's age (years)	20–29	23 (54.80%)	19 (45.20%)	0.477	0.788	
	30–39	42 (48.30%)	45 (51.70%)			1.82 (0.69–4.80)
	40–49	4 (50.00%)	4 (50.00%)			2.39 (0.41–14.21)
Mother's occupation	Self-employed	39 (48.80%)	41 (51.30%)	0.571	0.903	1.61 (0.38–6.66)
	Student	5 (62.50%	3 (37.50%)			0.62 (0.05–6.96)
	Employed	18 (51.40%)	17 (48.60%)			1.08 (0.22–5.20)
	Unemployed	7 (50.00%)	7 (50.00%)			
Mother's education	Primary	5 (41.70%)	7 (58.30%)	0.479	0.787	
	Secondary	31 (52.50%)	28 (47.50%)			0.88 (0.19–4.18)
	Tertiary	33 (50.00%)	33 (50.00%)			0.66 (0.13–3.40)
Neonates' sex	Female	36 (56.30%)	28 (43.80%)	1.664	0.197	
	Male	33 (45.20%)	40 (54.80%)			2.36 (1.01–5.54)^*∗*^
Neonate's weight (g)	600–999	0 (0.00%)	6 (100.00%)	32.428	0.001^*∗*^	
	1000–1499	1 (4.30%)	22 (95.70%)			
	1500–2499	68 (63.00%)	40 (37.00%)			

*χ* ^2^: chi square, ^*∗*^: significant (*p* < 0.05), OR: odd ratio.

## Data Availability

The data are not available due to ethical concerns.

## Abbreviations

MCHA: Mother and Child Hospital Akure
DAMA: Discharged against medical advice
NNS: Neonatal sepsis
FTT: Failure-to-Thrive
ELBW: Extremely low birth weight
VLBW: Very low birth weight
SBA: Severe birth asphyxia
NEC: Necrotizing enterocolitis
SGA: Small for gestational age
NNJ: Neonatal jaundice
NNT: Neonatal tetanus
HIE: Hypoxic ischemic encephalopathy
RDS: Respiratory distress syndrome
PROM: Premature rupture of membranes
NNEC: Neonatal necrotizing enterocolitis
HDN: Haemorrhagic disease of the new born
RVS: Retroviral disease.
